The article "Bioinformatics Analysis Reveals the Biomarker Value and Potential Mechanism of miR-675-3p in Gastric Cancer" was retracted in 2023. Reasons: signs of a paper mill; compromised peer review; unreliable results or conclusions.

# Bioinformatics Analysis Reveals the Biomarker Value and Potential Mechanism of miR-675-3p in Gastric Cancer

**DOI:** 10.1155/2022/5456554

**Published:** 2022-06-29

**Authors:** Ruyi Chen, Yi Li, Wei Ouyang, Shaoji Chen

**Affiliations:** ^1^Department of Gastrointestinal, The First Affiliated Hospital of Soochow University, Suzhou 215006, Jiangsu Province, China; ^2^Department of Otolaryngology, The First Affiliated Hospital of Soochow University, Suzhou 215006, Jiangsu Province, China; ^3^Department of Oncology, The First Affiliated Hospital of Soochow University, Suzhou 215006, Jiangsu Province, China

## Abstract

**Background:**

Gastric cancer (GC) is still the main challenge for the social and clinical system. Increasing studies have proved that microRNA dysfunction is closely associated with the GC progression. miR-675-3p has been confirmed as the tumor support in multiple tumor cells, while its role in GC remains unclear. Methods. The clinical data in the TCGA database were excavated for analyzing the role of miR-675-3p in pan-cancer and GC. qRT-PCR was applied to detect the abundances of the genes. The Starbase 2.0 was executed to target the prediction of miR-675-3p. Moreover, the enrichment analysis was performed with the DAVID database. The PPI-network analysis of the targets was performed with Cytoscape.

**Results:**

miR-675-3p was dramatically upregulated in multiple types of cancer, and elevated miR-675-3p was also found in GC tissues. Moreover, increased miR-675-3p was closely related with the poor survival rates of the patients. The qRT-PCR showed that miR-675-3p was extremely upregulated in GC tissues and cell lines. The enrichment analysis showed that the targets of miR-675-3p were located in the cellular nucleus and associated with the transcriptional misregulation in cancer. The PPI-network showed that three clusters and total of 40 genes were screened as potential hub nodes. Moreover, BRIP1, MYO5B, and PDS5B were related with the prognostic survival of the patients according to the TCGA database and decreased BRIP1, MYO5B, and PDS5B were also found in GC cell lines.

**Conclusion:**

This study identified miR-675-3p as a potential biomarker in GC development and revealed the potential regulation network of miR-675-3p.

## 1. Introduction

Gastric cancer (GC) is a prevalent malignant disease in modern society, which also occupies a considerable proportion in cancer-related death. The increasing number of patients have been diagnosed with gastric cancer every year [1, 2]. Although the current medicine strategies such as surgery, chemotherapy, and radiotherapy have been effectively blocked the deterioration of the symptom, this disease is still far from completed healing [3, 4]. Considerable patients still exhibit poor outcomes and low survival rates in long term prognosis. In the past decade, an increasing number of reporters have gradually revealed the pathological mechanism of GC formation and development [5]. However, more biomarkers and related regulation mechanisms are still urgent for further improvement of GC diagnosis and intervention.

The article "Bioinformatics Analysis Reveals the Biomarker Value and Potential Mechanism of miR-675-3p in Gastric Cancer" was retracted in 2023. Reasons: signs of a paper mill; compromised peer review; unreliable results or conclusions.

MicroRNAs (miRNAs) play pivotal roles in cellular metabolism, and the disorder of miRNAs profile has also been widely accepted as a direct reason [6]. For cancer development, the aberrant profiles of microRNA have been confirmed as a biomarker event [7, 8]. For GC, abundant pieces of evidence have showed that the miRNA profile in the serums of the patients generally exhibit remarkable differences compared with the healthy persons, and some miRNA also deriving the deterioration of the symptoms [9]. Therefore, miRNAs have been gradually recognized as the promising targets for the clinical diagnosis and drug development [10, 11]. Moreover, the change in the regulation network consisted with miRNAs and the related mRNAs is also closely associated with the malignant progression of GC [12]. Several reporters have indicated that miR-675-3p serves as an oncogene in some types of cancer, while few studies have revealed the role and related mechanism of miR-675-3p in GC [13]. The bioinformatics analysis based on the excavation of microarray datasets have been confirmed as a useful method in investigating the molecular regulation of multiple diseases [14].

This study was conducted to investigate the association of miR-675-3p and GC and reveal the related potential molecular mechanism in the progression of GC via excavating the TCGA database and thus provide some valuable references for the diagnosis and treatment of GC.

## 2. Materials and Methods

### 2.1. The Clinical Data Analysis of TCGA

The clinical data of the patients with GC were originated from The Cancer Genome Atlas (TCGA) database. The expression of miR-675-3p in GC and pan-cancer were analyzed and visualized with R language. The survival curves of the genes were also analyzed and visualized by R language. Besides, the difference of the abundance of the proteins in tumor and normal tissues were analyzed with the GEPIA database (http://gepia.cancer-pku.cn/).

### 2.2. Clinical Tissues

The clinical tissues including tumor tissues and adjacent tissues were originated from the donation of the hospital, and the study were approved by the ethics committee of the hospital.

### 2.3. Cell Culture

The GC cell lines including BGC-823, SGC-7901, and MGC-803, and human normal cell line GES-1 were purchased from Tongpai Biotechnology Co. Ltd, Shanghai, China. The cells were cultured in an incubator containing 5% CO_2_ with a constant temperature condition of 37°C. The DMEM was selected as the culture medium, and 10% FBS was used for maintaining cells growth.

The article "Bioinformatics Analysis Reveals the Biomarker Value and Potential Mechanism of miR-675-3p in Gastric Cancer" was retracted in 2023. Reasons: signs of a paper mill; compromised peer review; unreliable results or conclusions.

### 2.4. Real-Time Quantitative Reverse Transcription PCR

The extraction of total RNA in the tissues or cells were performed by TRIzol reagent (Shanghai Crystal Biological Engineering Co. Ltd, Shanghai, China), and then the related concentrations were detected with BCA kits. Subsequently, the PrimeScript RT-PCR kit (Shanghai Shanran Biotechnology Co. Ltd, Shanghai, China) was executed to cDNA reverse transcription. After that, the cDNAs were used for measuring the abundance of the genes. For reaction conditions: 95°C for 5 min, followed by 40 cycles of 95°C for 15 s, 62°C for 30 s, and 72°C for 30 s. Finally, the 2−(ΔΔCt) method was applied to calculate the related abundances of the genes. The primer information was listed in Table 1.

### 2.5. Gene Ontology (GO) Enrichment Analysis

The Starbase 2.0 database was applied to predict the targets of miR-675-3p. Subsequently, the DAVID database was executed to GO enrichment analysis of the targets. In brief, the symbol names of the targets were uploaded on DAVID, and then the targets were analyzed by functional annotation. After that, the related results including the Cellular Components (CCs), Biological Process (BP), and Molecular Function (MF) of the genes were obtained from the database. Besides, the visualization of the results was analyzed with R language.

### 2.6. Kyoto Encyclopedia of Genes and Genomes (KEGG) Enrichment Analysis

KEGG enrichment analysis of the targets were performed by the DAVID database. Briefly, the symbol names of the targets were uploaded on DAVID, and then the targets were analyzed by functional annotation. After that, the KEGG enrichment were obtained from the database.

### 2.7. Network Analysis

The STRING database was executed to the protein-protein interaction (PPI) network analysis of the targets [15]. Briefly, the targets were uploaded to the STRING database, and then the related results were obtained from the database. Besides, the visualization of the results was performed by Cytoscape.

### 2.8. Data Analysis

The experiments in this study were repeated three times at least. The SPSS 20.0 was executed to data analysis. The methods including the Chi-squared test or ANOVA with Tukey's posthoc-test were applied to analyze the difference in the data. Besides, ^∗∗^*P* < 0.05 represented that the difference had statistical significance.

## 3. Results

### 3.1. The Abundance of miR-675-3p in Pan-Cancer Were Analyzed by TCGA Database

The abundance profile of miR-675-3p was investigated in pan-cancer according to the TCGA database. The results showed that miR-675-3p was significantly upregulated in multiple types of cancer, especially in GC. It implied the promoter role of miR-675-3p in cancer (Figures 1(a)& 1(c)). Moreover, it was found that increased miR-675-3p was related with the poor prognosis of the patients with GC (Figure 1(b)).

The article "Bioinformatics Analysis Reveals the Biomarker Value and Potential Mechanism of miR-675-3p in Gastric Cancer" was retracted in 2023. Reasons: signs of a paper mill; compromised peer review; unreliable results or conclusions.

### 3.2. Increased miR-675-3p Was Detected in GC Tissues and Cell Lines

To provide more actual pieces of evidence, the pathological tissues and normal tissues of the GC patients were used to detect the abundance of miR-675-3p in clinical pathological samples. The results showed that miR-675-3p was obviously upregulated in the tumor tissues compared with the related adjacent tissues (Figure 2(a), *P* < 0.01). Moreover, increased miR-675-3p was also found in the GC cells lines (Figure 2(b), *P* < 0.01). These proofs suggested that miR-675-3p upregulation is a biomarker event in GC development.

### 3.3. Function and Pathway Analysis

To illustrate the potential roles and related functional mechanism of miR-675-3p, the targets of miR-675-3p were predicted by the Starbase database, and the targets were analyzed with the DAVID database. The GO enrichment showed that the targets of miR-675-3p were mainly enriched in the cellular nucleus, cytoplasm, cytosol, and nucleoplasm. The targets were involved in the regulation of transcription, gene expression, and protein phosphorylation and also took part in the regulation of cellular proliferation and cycle. Moreover, it was found that the targets were associated with protein binding, metal ion binding, RNA/DNA binding, etc. (Figure 3(a), *P* < 0.01). The KEGG enrichment showed that the targets were associated with transcriptional misregulation in cancer, and the genes including MEF2C, CCNT2, BCL11 B, PBX3, MLLT3, KLF3, FLI1, HOXA11, IGF1R, ELK4, MEIS1, NR4A3, SIX4, NSD2, and REL were enriched in this cellular pathway (Figure 3(b), *P* < 0.01).

### 3.4. Network Analysis

The targets of miR-675-3p were analyzed with PPI-network. The results showed that three clusters including cluster 1 with 16 nodes and 60 edges, cluster 2 with 8 nodes and 24 edges, and cluster 3 with 16 nodes and 50 edges (Figure 4). For cluster 1, FMR1, SRSF2, DDX3X, SKIV2L2, CAMK2D, and TIAL1 were screened as hub nodes (Figure 4(a)). For cluster 2, EIF4E and IGF1R were screened as hub nodes (Figure 4(b)). For cluster 3, TFRC and PI3KC2A were screened as the hub nodes (Figure 4(c)).

### 3.5. The Expression Profile and Prognostic Value of the Hub Nodes in GC

The hub nodes were analyzed with the TCGA database to identify the valuable targets. The results showed that reduced BRIP1, MYO5B, and PDS5B were related with poor survival rates (Figure 5(a)–5(d), *P* < 0.01). Moreover, the qRT-PCR showed that BRIP1, MYO5B, PDS5B, and STAG1 were dramatically downregulated in GC cell lines (Figure 6(a)–6(d), *P* < 0.01).

The article "Bioinformatics Analysis Reveals the Biomarker Value and Potential Mechanism of miR-675-3p in Gastric Cancer" was retracted in 2023. Reasons: signs of a paper mill; compromised peer review; unreliable results or conclusions.

## 4. Discussion

The intervention on gastric cancer (GC) has been continually focused on by many medical and academic institutions. Although it has been achieved great accomplishments in the prevention and therapy of GC, this disease remains the main challenge for the public health system in most countries due to its poor prognosis [16, 17]. Noncoding RNAs such as miRNAs have been confirmed to involve the regulation mechanism in the progression of GC and thus have great potential in drug development and clinical diagnosis [18]. Bioinformatics excavation and analysis has been confirmed as an effective strategy for revealing potential biomarkers and related mechanism [19]. This study investigated the connection of miR-675-3p and GC development and revealed the potential regulation mechanism via the excavation of a public database.

miRNA dysfunction has been widely accepted as a general event in cancer development. For GC, accumulating reporters have indicated that some miRNAs directly influence the malignant behaviors of GC cells and thus promote the cancer deterioration [20, 21]. In this research, it was confirmed that miR-675-3p was dramatically upregulated in multiple types of cancer. Wang et al. have indicated that miR-675-3p could promote the epithelial-mesenchymal transition of pancreatic cancer cells [22]. Thus, it implies that miR-675-3p upregulation is a common event in cancer development. Besides, increased miR-675-3p was related with the low survival rates of the patients with GC according to the TCGA database. Elevated miR-675-3p has been observed in multiple types of cancer. Moreover, miR-675-3p has also been identified as a valuable biomarker for the prognostic prediction of the patients with melanoma [13]. Thus, it is supported that miR-675-3p was a potential biomarker in GC development.

The dysfunction of the cellular pathway has been generally confirmed in cancer development. miRNAs have been widely recognized as the regulators for cellular phenotype depending on their molecular functions [23]. miR-675-3p has been proved to drive the malignant progression of pancreatic cancer via influencing the STAT3 pathway [22]. For GC, various reports have confirmed that the aberrant abundance of miRNA is related with the progression of cancer via influence the cellular signal transduction. The aberrant activities of the pathways such as PI3K/AKT and Wnt/*β*-catenin can directly induce the malignant phenotype of tumor cells, including proliferation, antiapoptosis [6, 24]. In this study, the targets of miR-675-3p were enriched in the transcriptional misregulation in cancer. Moreover, the targets of miR-675-3p were mainly located in the cellular nucleus, involved in the regulation of transcription, and also took part in the regulation of cellular proliferation and cycle. The KEGG enrichment showed that the targets were associated with transcriptional misregulation in cancer.

miRNAs functions as regulators for protein translation via combining with the related mRNAs, and the dysfunction of the miRNA-mRNA network has also been attributed as a direct reason of GC [25, 26]. In this study, the 40 genes in the targets of miR-675-3p were screened as the hub nodes. It was found that reduced BRIP1, MYO5B, and PDS5B are related with the low survival rates of the patients with GC. BRIP1 mutation may be a potential reason inducing the progression of breast cancer, and significant BRIP1 mutation has also been predicted with an increased risk of ovarian cancer [27, 28]. This study also found that BRIP1 was dramatically downregulated in GC cell lines, suggesting the decreased BRIP1 is a biomarker event in GC development. MYO5B is a member of nonfilamentous myosins, which takes part in intracellular transport via depending on actin [29]. The study has indicated that MYO5B serves as a tumor inhibitor in GC cells, and the inactivation of MYO5B could induce the invasion of GC cells [30]. This study also confirmed that MYO5B was extremely reduced in GC cell lines, which suggests that MYO5B is a biomarker in GC progression. PDS5B serves as a pivotal role in maintaining the stabilization of the replication fork, and it is also involved in the DNA repair [33]. PDS5B dysfunction is also associated with cancer development. The antitumor effect of PDS5B in multiple tumors has been confirmed by several reports. Xu et al. have revealed that PDS5B is obviously decreased in lung cancer cells and increased PDS5B can effectively impede the malignant proliferation and invasion of the tumor cells [34]. This study also confirmed that PDS5B was remarkably downregulated in GC cells.

The article "Bioinformatics Analysis Reveals the Biomarker Value and Potential Mechanism of miR-675-3p in Gastric Cancer" was retracted in 2023. Reasons: signs of a paper mill; compromised peer review; unreliable results or conclusions.

## 5. Conclusion

This study revealed that miR-675-3p is a biomarker in GC development, and it has potential value in clinical research and therapy of GC.

## Figures and Tables

**Figure 1:** miR-675-3p was obviously upregulated in multiple tumors especially in GC (A) The abundance of miR-675-3p in pan-cancer. (B)-(C) The expression and survival curve of miR-675-3p in GC.

**Figure 2:** miR-675-3p was obviously upregulated in GC tissues and cell lines. (a) The abundance of miR-675-3p in GC tissues. (b) The abundance of miR-675-3p in GC cell lines.

**Figure 3:** The enrichment analysis for the targets of miR-675-3p. (a) GO enrichment analysis. (b) KEGG enrichment analysis.

**Figure 4:** The PPI-network analysis for the targets of miR-675-3p. (A)-(C) Cluster 1, Cluster 2, and Cluster 3 were analyzed with Cytoscape.

**Figure 5:** The connections of the screened targets and the survival rate of patients according to the TCGA database. (A)-(D) The survival curves of BRIP1, MYO5B, PDS5B, and STAG1.

**Figure 6:** The abundances of the screened targets in GC cell lines. (A)-(D) The abundances of BRIP1, MYO5B, PDS5B, and STAG1 in GC cell lines.

**Table 1:** Primer information.

Name of primer	Sequences
miR-675-3p-F	5′-GCCGAGCATCTTACCGGACGT-3′
miR-675-3p-R	5′-CTCAACTGGTGTCGTGGA-3′
BRIP1-F	5′-TAAGAGCTTACCACCGCTGC-3′
BRIP1-R	5′-GTGGCTGCTCTCCTGACATT-3′
MYO5B-F	5′-TCGGGGTCCTGGACATCTAT-3′
MYO5B-R	5′- CCAGTTTGAAAACATGCGAGTTG-3′
PDS5B-F	5′-TCCACACAGTCCACACCAC-3′
PDS5B-R	5′-ATCATTTTCCTTAGTAGCTGC-3′
STAG1-F	5′-CGTACCTGCAGCACGAGAT-3′
STAG1-R	5′-CCTGGCACTATCCATCAGGT-3′
U6-F	5′-CTCGCTTCGGCAGCACA-3′
U6-R	5′-AACGCTTCACGAATTTGCGT-3′

## Data Availability

The data used to support the findings of this study are available from the corresponding author upon request.

## References

[1] Shiotani A., Cen P., Graham D. Y. (2013). Eradication of gastric cancer is now both possible and practical. *Seminars in Cancer Biology*.

[2] Mahipal A., Choi M., Kim R. (2015). Second-line treatment of advanced gastric cancer: where do we stand?. *Journal of the National Comprehensive Cancer Network*.

[3] Shitara K., Ohtsu A. (2016). Advances in systemic therapy for metastatic or advanced gastric cancer. *Journal of the National Comprehensive Cancer Network*.

[4] Yu J., Zhang Y., Leung L.-H., Liu L., Yang F., Yao X. (2016). Efficacy and safety of angiogenesis inhibitors in advanced gastric cancer: a systematic review and meta-analysis. *Journal of Hematology & Oncology*.

[5] Talley N. J., Fock K. M., Moayyedi P. (2008). Gastric cancer consensus conference RecommendsHelicobacter pyloriScreening and treatment in asymptomatic persons from high-risk populations to prevent gastric cancer. *American Journal of Gastroenterology*.

[6] Deng P., Li K., Gu F. (2021). LINC00242/miR-1-3p/G6PD axis regulates Warburg effect and affects gastric cancer proliferation and apoptosis. *Molecular Medicine*.

[7] Feng Q., Wu X., Li F. (2017). miR-27b inhibits gastric cancer metastasis by targeting NR2F2. *Protein & Cell*.

[8] Yang X.-Z., Cheng T.-T., He Q.-J. (2018). LINC01133 as ceRNA inhibits gastric cancer progression by sponging miR-106a-3p to regulate APC expression and the Wnt/*β*-catenin pathway. *Molecular Cancer*.

The article "Bioinformatics Analysis Reveals the Biomarker Value and Potential Mechanism of miR-675-3p in Gastric Cancer" was retracted in 2023. Reasons: signs of a paper mill; compromised peer review; unreliable results or conclusions.

[9] Iqbal M. A., Arora S., Prakasam G., Calin G. A., Syed M. A. (2019). MicroRNA in lung cancer: role, mechanisms, pathways and therapeutic relevance. *Molecular Aspects of Medicine*.

[10] Fabris L., Ceder Y., Chinnaiyan A. M. (2016). The potential of MicroRNAs as prostate cancer biomarkers. *European Urology*.

[11] Zhang J., Liu H., Hou L. (2017). Circular RNA_LARP4 inhibits cell proliferation and invasion of gastric cancer by sponging miR-424-5p and regulating LATS1 expression. *Molecular Cancer*.

[12] Zhang Z., Pi J., Zou D. (2019). microRNA arm-imbalance in part from complementary targets mediated decay promotes gastric cancer progression. *Nature Communications*.

[13] Zhao C.-C., Guo H., Wang Y., Li J.-H. (2021). Comprehensive upstream and downstream regulatory analyses identify miR-675-3p as a potential prognostic biomarker in melanoma. *Human Cell*.

[14] Zhang K., Zhang L., Mi Y. (2020). A ceRNA network and a potential regulatory axis in gastric cancer with different degrees of immune cell infiltration. *Cancer Science*.

[15] Cao M., Pietras C. M., Feng X. (2014). New directions for diffusion-based network prediction of protein function: incorporating pathways with confidence. *Bioinformatics*.

[16] Olino K., Park T., Ahuja N. (2020). Exposing Hidden Targets: combining epigenetic and immunotherapy to overcome cancer resistance. *Seminars in Cancer Biology*.

[17] Liu J., Li Z., Teng W., Ye X. (2020). Identification of downregulated circRNAs from tissue and plasma of patients with gastric cancer and construction of a circRNA-miRNA-mRNA network. *Journal of Cellular Biochemistry*.

[18] Zhang J.-X., Xu Y., Gao Y. (2017). Decreased expression of miR-939 contributes to chemoresistance and metastasis of gastric cancer via dysregulation of SLC34A2 and Raf/MEK/ERK pathway. *Molecular Cancer*.

[19] Ziyu N., Chenchen F., Chao S. (2019). Corrigendum to: topologically inferring active miRNA-mediated subpathways toward precise cancer classification by directed random walk. *Mol Oncol*.

[20] Shin V. Y., Ng E. K. O., Chan V. W., Kwong A., Chu K.-M. (2015). A three-miRNA signature as promising non-invasive diagnostic marker for gastric cancer. *Molecular Cancer*.

[21] Jiang Y., Jin S., Tan S., Shen Q., Xue Y. (2019). MiR-203 acts as a radiosensitizer of gastric cancer cells by directly targeting ZEB1. *OncoTargets and Therapy*.

[22] Wang F., Rong L., Zhang Z. (2020). LncRNA H19-derived miR-675-3p promotes epithelial-mesenchymal transition and stemness in human pancreatic cancer cells by targeting the STAT3 pathway. *Journal of Cancer*.

[23] Qi H., Xiao Z., Wang Y. (2019 Aug). Long non-coding RNA LINC00665 gastric cancer tumorigenesis by regulation miR-149-3p/RNF2 axis. *OncoTargets and Therapy*.

The article "Bioinformatics Analysis Reveals the Biomarker Value and Potential Mechanism of miR-675-3p in Gastric Cancer" was retracted in 2023. Reasons: signs of a paper mill; compromised peer review; unreliable results or conclusions.

[24] Huang Y., Zhang J., Hou L. (2017). LncRNA AK023391 promotes tumorigenesis and invasion of gastric cancer through activation of the PI3K/Akt signaling pathway. *Journal of Experimental & Clinical Cancer Research*.

[25] De Nicolo A., Tancredi M., Lombardi G. (2008). A novel breast cancer-associated BRIP1 (FANCJ/BACH1) germ-line mutation impairs protein stability and function. *Clinical Cancer Research*.

[26] Rafnar T., Gudbjartsson D. F., Sulem P. (2011). Mutations in BRIP1 confer high risk of ovarian cancer. *Nature Genetics*.

[27] Kravtsov D., Mashukova A., Forteza R., Rodriguez M. M., Ameen N. A., Salas P. J. (2014). Myosin 5b loss of function leads to defects in polarized signaling: implication for microvillus inclusion disease pathogenesis and treatment. *American Journal of Physiology - Gastrointestinal and Liver Physiology*.

[28] Dong W., Chen X., Chen P., Yue D., Zhu L., Fan Q. (2012). Inactivation of MYO5B promotes invasion and motility in gastric cancer cells. *Digestive Diseases and Sciences*.

[29] Morales C., Ruiz-Torres M., Rodríguez-Acebes S. (2020). PDS5 proteins are required for proper cohesin dynamics and participate in replication fork protection. *Journal of Biological Chemistry*.

[30] Xu H., Zhou W., Zhang F. (2021). PDS5B inhibits cell proliferation, migration, and invasion via upregulation of LATS1 in lung cancer cells. *Cell Death Discovery*.

